# Association between *TLR*-9 gene rs187084 polymorphism and knee osteoarthritis in a Chinese population

**DOI:** 10.1042/BSR20170844

**Published:** 2017-10-17

**Authors:** Mingfeng Zheng, Shiyuan Shi, Qi Zheng, Yifan Wang, Xiaozhang Ying, Yanghui Jin

**Affiliations:** Department of Orthopedics, Hangzhou Red Cross Hospital (Zhejiang Chinese Medicine Integrated Hospital), 208 Huanchengdong Road, Hangzhou, Zhejiang 310003, China

**Keywords:** bioinformatics, knee osteoarthritis, rs187084 polymorphism, Toll-like receptor 9

## Abstract

Osteoarthritis (OA) is a complex disease that is induced by many genetic risk variants and other factors. To examine the role of toll-like receptor 9 (TLR-9) in OA patients, we conducted a case–control study involving 215 knee OA (KOA) patients and 215 controls in a Chinese population. Genotyping with a custom-by-design 48-Plex single nucleotide polymorphism Scan™ Kit showed the *TLR*-9 gene rs187084 polymorphism was associated with an increased risk of KOA. Stratification analyses further validated this finding among old people (age ≥ 55 years). In conclusion, *TLR*-9 gene rs187084 polymorphism is positively correlated with susceptibility to KOA, especially among old people. Nevertheless, this finding should be confirmed by larger size studies with more ethnic populations.

## Introduction

Osteoarthritis (OA) is a degenerative joint disease characterized by joint destruction with cartilage loss and occasional gross derangement of joint integrity [1]. Knee osteoarthritis (KOA) causes the most severe economic and psychological burdens because pains in weight-bearing joints often need surgical intervention [2]. Although the etiology of KOA remains unclear, previous evidence show aging, obesity, history of injury, and smoking habit are all associated with risks of KOA [3]. Notably, genetic factors account for 50% of the risk of OA development [4,5]. Therefore, candidate gene studies may provide insight about OA development.

Toll-like receptors (TLR) could bind to various damage-associated molecular patterns, which may be associated with autoinflammation and the production of costimulatory signals necessary for adaptive immune reactions [6]. TLR-9 is located on chromosome 3p21.2 and has two exon counts. Stimulation of TLR-9 by its ligands triggers a signaling pathway common for all TLRs, resulting in activation of nuclear factor-κB (NF-κB) transcription factor and production of proinflammatory cytokines, including tumor necrosis factor-α and interleukin-6 [7]. These proinflammatory cytokines are positively correlated with cartilage degradation in OA [8,9]. Macrophages and their products contribute to the induction of OA triggered by bacterial DNA [10]. These observations suggest TLR-9 may affect the development of OA.

In 2011, a two-stage case–control study with 503 OA patients and 428 controls from Taiwan revealed that the risk of OA in a Chinese population was intensified by *TLR*-9 gene rs187084 polymorphism and associated with T allele or TT genotype of this polymorphism [11]. Balbaloglu et al. [12] replicated a positive finding in a Turkish population, but the risk of KOA was increased by the CC genotype rather than the T allele or TT genotype of rs187084 polymorphism. Regarding the conflicting findings of these studies, we conducted this hospital-based case–control study to investigate and validate the association between *TLR*-9 gene rs187084 polymorphism and KOA risk in a Chinese population.

## Patients and methods

### Study population

Totally, 215 KOA patients and 215 healthy controls were consecutively recruited from Hospital of Integrated Traditional Chinese and Western Medicine (Hangzhou Red Cross Hospital) in Zhejiang Province between September 2013 and December 2016. The diagnosis of KOA fulfilled the American College of Rheumatology criteria (1987) [13] and included primary OA with any symptom and radiographic sign of OA according to the Kellgren–Lawrence (K–L) grading system. Two investigators blind to the clinical information examined the radiographs of each participant and obtained a global K–L score (0–4 scale) by an atlas of radiographic features. Patients with any systemic inflammatory or autoimmune disorder, or any type of malignant or chronic illness were excluded from the present study. The controls had no personal or family history of KOA and were matched for age (± 5 years) and sex.

This case–control study was approved by the Ethics Committee of our Hospital and performed according to ‘Declaration of Helsinki’. All patients provided written informed consent prior to participation.

### Functional enrichment analysis and single nucleotide polymorphism (SNP) selection

Functional protein association network establishment and functional enrichment analysis were conducted on String (http://www.string-db.org/). Only significant ‘Kyoto Encyclopedia of Genes and Genomes’ (KEGG) pathways with *P*≤0.05 and number of enriched genes ≥ 3 were concerned. We explored whether *TLR*-9 gene polymorphisms were in strong linkage disequilibrium (LD) or independently contributed to the susceptibility of KOA, and whether they can capture additional significant variants on Haploview 4.2 (Broad Institute of MIT and Harvard, U.S.A).

### Genotyping

From each patient, 2 ml of peripheral blood was collected in a test tube containing ethylenediaminetetraacetic acid, and sent to genomic DNA extraction on a QIAamp DNA Blood Mini Kit (Qiagen, Hilden, Germany) according to the manufacturer’s instruction. Single nucleotide polymorphism (SNP) genotyping was performed using a custom-by-design 48-Plex SNP scan^TM^ Kit (Genesky Biotechnologies Inc., Shanghai, China).

### Statistical analysis

The demographic and clinical characteristics of the study population were evaluated via chi-squared test. Association between *TLR*-9 gene rs187084 polymorphism and KOA risk was assessed by logistic regression with odds ratio (OR) and 95% confidence interval (CI). The most common homozygote was considered as a reference. Hardy–Weinberg equilibrium for genotype distribution of rs187084 polymorphism in controls was tested by goodness-of- fit chi-squared test. All statistical analyses were performed on SAS 9.1.3 (SAS Institute, Cary, NC, U.S.A.) with the significant level at *P*<0.05.

## Results

### Bioinformatics analysis

Figure 1 shows a functional protein association network of TLR-9. Protein-related genes can interact to large degree. Genes positively correlated with TLR-9 include Bruton tyrosine kinase (BTK), CD40 molecule, myeloid differentiation primary response 88 (MYD88), and interleukin 1 receptor associated kinase 1 (IRAK1). Gene enrichment analysis by considering KEGG pathways shows that most of these genes were enriched in the NF-κB pathway and the TLR pathway. The details of KEGG pathways were summarized in Table 1. As reported, Barton et al. [7] have demonstrated that all TLRs activate MYD88-dependent pathways (NF-κB, mitogen-activated protein kinases, extracellular signal-regulated kinase, p53, and c-Jun N-terminal kinase) to induce a cure set of stereotyped responses, such as inflammation. Our bioinformatics analysis is consistent with this finding to some extent. Therefore, TLR-9 may activate the NF-κB pathway and thereby contributes to inflammation, a main manifestation of OA.

**Figure 1:** A functional protein association network for TLR-9 Known interactions (light blue and purple line), predicted interactions (green, red, and navy blue line), and others (yellow, black, and gray line)

**Table 1:** KEGG enrichment analysis for *TLR*-9 related genes

Pathway ID	Pathway description	Gene count	Gene symbol
4064	NF-kappa B signaling pathway	5	BTK, CD40, IRAK1, IRAK4, MYD88
4620	Toll-like receptor signaling pathway	5	CD40, IRAK1, IRAK4, MYD88, TLR-9
5152	Tuberculosis	5	IRAK1, IRAK4, ITGAX, MYD88, TLR-9
5142	Chagas disease	4	IRAK1, IRAK4, MYD88, TLR-9
5145	Toxoplasmosis	4	CD40, IRAK1, IRAK4, MYD88
5162	Measles	4	IRAK1, IRAK4, MYD88, TLR-9
5144	Malaria	3	CD40, MYD88, TLR-9
5133	Pertussis	3	IRAK1, IRAK4, MYD88
5140	Leishmaniasis	3	IRAK1, IRAK4, MYD88
4210	Apoptosis	3	IRAK1, IRAK4, MYD88

Abbreviations: BTK, Bruton’s tyrosine kinase; CD40, CD40 molecule; IRAK1, interleukin 1 receptor associated kinase 1; IRAK4, interleukin 1 receptor associated kinase 4; MYD88, myeloid differentiation primary response 88.

After determination of functional genes, tagger SNPs were screened on Haploview 4.2. Relevant parameters were set as follows: HW *P*-value cutoff = 0.001; min. genotype = 75%; Max# mendel error = 1; Minimum allele frequency (MAF) = 0.05. Three tagger SNPs (rs351240, rs352139, and rs187084) were identified, two of which (rs352139 and rs187084) were in LD (Figure 2). According to 1000 Genomes Browser, rs352139 has higher MAF than rs187084 (0.49 vs. 0.38). However, rs352139 and rs187084 polymorphisms are located on in the intron region and promoter region of *TLR*-9 gene respectively. TLR-9 rs187084 polymorphism may affect its binding to transcription factors, which might indirectly contribute to the development of KOA. Therefore, only rs187084 polymorphism was involved in the analyses.

**Figure 2:** Linkage disequilibrium for *TLR*-9 gene

### Clinical information of the study population

Table 2 lists the clinical information of the patients. The subjects were fully matched for age and sex (*P*=0.593 and *P*=0.328 respectively). A significant association was found in the subgroup of body mass index (BMI). In addition, disease severity in the KOA cases and controls was assessed via the K–L grading. The controls and cases were concentrated in grade 0–1 and grade 2–4 respectively.

**Table 2:** Patient demographics and risk factors in knee osteoarthritis

Variable	Cases (*n*=215)	Controls (*n*=215)	*P*
Age (years)			
≤50	104	99	0.593
>50	111	116	
Sex			
Female	130(60.5%)	120(55.8%)	0.328
Male	85(39.5%)	95(44.2%)	
Body mass index	26.2 ± 3.4	24.6 ± 3.7	<0.001
Kellgren–Lawrence grading			
0	–	137(63.7%)	
1	–	78(36.3%)	
2	54(25.1%)	–	
3	105(48.8%)	–	
4	56(26.0%)	–	

### Association between *TLR*-9 gene rs187084 polymorphism and KOA risk

The genotyping frequencies of *TLR*-9 gene rs187084 polymorphism in cases and controls were summarized in Table 3. The genotype distribution in the controls conformed to Hardy–Weinberg equilibrium (*P*=0.183). The subjects with CC genotype versus TT genotype of rs187084 polymorphism have a significantly increased risk of KOA (OR 1.96, 95% CI, 1.01–3.82, *P*=0.048). Moreover, C allele of rs187084 polymorphism is positively correlated with the risk of KOA (C vs. T, OR 1.34, 95% CI, 1.01–1.78, *P*=0.043). No significant association between TLR-9 rs187084 polymorphism and the risk of KOA was found in the recessive model (*P*=0.109) or the dominant model (*P*=0.075).

**Table 3:** Logistic regression analysis of associations between TLR-9 rs187084 polymorphism and risk of osteoarthritis

Genotype	Cases* (*n*=215)		Controls* (*n*=215)		OR (95% CI)	*P*
	*n*	%	*n*	%		
TC vs. TT	107/73	49.8/34.0	101/92	47.0/42.8	1.34 (0.89–2.01)	0.167
CC vs. TT	28/73	13.0/34.0	18/92	8.4/42.8	**1.96 (1.01–3.82)**	0.048
CC vs. TC vs. TT						
TC+CC vs. TT	135/73	62.8/34.0	119/92	55.4/42.8	1.43 (0.96–2.12)	0.075
CC vs. TC + TT	28/180	13.0/83.7	18/193	8.4/89.8	1.67 (0.89–3.12)	0.109
C vs. T	163/253	37.9/58.8	137/285	31.9/66.3	**1.34 (1.01–1.78)**	0.043

* The genotyping was successful in 208 cases and 211 controls.

Bold values are statistically significant (*P*<0.05).

Stratified analyses of sex and age are illustrated in Table 4. For old participants (age ≥ 55 years), the CC genotype of rs187084 polymorphism increased the risk of KOA by 3.34-fold compared with the TT genotype. Old subjects carrying the CC genotype had a significantly higher risk of KOA than those carrying the TC + TT genotypes (OR 2.61, 95% CI, 1.08–6.33, *P*=0.034). However, no significant association was observed in the stratified analysis of sex.

**Table 4:** Stratified analyses between TLR-9 rs187084 polymorphism and the risk of osteoarthritis

Variable	TLR-9 rs187084 (case/control)			CC vs. TT	CC+TC vs. TT	CC vs. TC+TT
	CC	TC	TT			
Sex						
Male	12/7	37/45	32/41	2.20 (0.78–6.23); 0.138	1.21 (0.66–2.21); 0.542	2.14 (0.80–5.72); 0.131
Female	16/11	70/56	41/51	1.81 (0.76–4.32); 0.182	1.60 (0.95–2.69); 0.078	2.61 (1.08–6.33); 0.415
Age (years)						
<55	11/10	54/48	38/37	1.07 (0.41–2.82); 0.890	1.09 (0.61–1.94); 0.766	1.02 (0.41–2.51); 0.972
≥55	17/8	53/53	35/55	**3.34 (1.30-8.56)**; 0.012	**1.80 (1.05–3.11)**; 0.034	**2.61 (1.08–6.33)**; 0.034

Bold values are statistically significant (*P*<0.05).

## Discussion

There is a wide consensus about the following two functions of TLRs: first, TLRs are associated with the activation of the innate and adaptive anti-infection host defense by recognizing microbe-associated molecular patterns; second, TLRs play important roles in autoinflammation and inflammatory factor production [6]. TLR-9 could recognize unmethylated CpG-rich and pathogen-derived DNA sequences [14] and increase the risk of autoimmune disease by stimulating B cells [15]. Remarkably, rs187084 polymorphism of *TLR*-9 gene was located in the promoter region, and Haploview screening found it was a tagger SNP. Therefore, the association between *TLR*-9 gene rs187084 polymorphism and relevant diseases has been widely investigated, such as systemic lupus erythematous (SLE) [16], OA [12], malaria [17], and sepsis [18]. Recently, TLR-9 overexpression was identified in SLE patients [19], which may stimulate B cells and induce SLE pathogenesis [20]. However, no article has directly uncovered the function of TLR-9 in the etiology of OA. After bioinformation analysis, we hypothesized that TLR-9 could activate NF-κB transcription factors to affect the production of proinflammatory cytokines, thus contributing to the development of OA. In addition, SNPs have been demonstrated to influence gene expression and function [21].

TLRs are essential molecules implicated in both innate and adaptive immune responses [22]. Many studies focused on the association between TLR-9 promoter polymorphism (rs187084) and autoimmune diseases, such as SLE [22], rheumatoid arthritis [23], and OA [12]. TLR-9 rs187084 polymorphism is associated weakly with SLE risk [22], but significantly with the risk of rheumatoid arthritis [23] or OA [12]. SLE is related to apoptosis abnormalities instead of inflammation, which is a core characteristic of rheumatoid arthritis or OA. KEGG pathway analysis suggests TLR-9 and its interacting genes are associated mostly with NF-κB pathway and TLR pathway, but weakly with apoptosis pathway. TLR-9 may play pathway-dependent roles, which might partly explain the association between TLR-9 rs187084 polymorphism and some autoimmune diseases.

In a two-stage case–control study with 503 patients and 428 controls, Su et al. [11] first investigated the association between TLR-9 rs187084 polymorphism and KOA risk in a Chinese population from Taiwan, and found through stage 1, stage 2, and combined stage analyses that T allele of rs187084 polymorphism was associated with the increased risk of OA. A case–control study with 272 cases and 296 controls in a Turkish population showed that CC genotype of rs187084 polymorphism had a higher risk of OA [12]. Our study with a Chinese population (215 cases and 215 controls) suggests C allele or CC genotype of rs187084 polymorphism is positively correlated with the increased risk of OA. Obviously, our study is different from Su et al. [11] on the identification of risk allele (C allele vs. T allele). We also found CC genotype increased the risk of OA, which was not reported by Su et al. [11], but was consistent with Balbaloglu et al. [12]. The C allele frequencies in the cases versus controls were as follows: 0.28 vs. 0.37 [11], 0.43 vs. 0.38 [12], and 0.39 vs. 0.32 (the present study). We hypothesize that the conflicting findings of the above studies may be attributed to the different gene distributions of these ethnicities, and also to genetic heterogeneity of OA in different populations, clinical heterogeneity and different sample sizes. To our knowledge, this is the first case–control study to address the association between *TLR*-9 gene rs187084 polymorphism and OA risk in a Chinese population from mainland China. The stratified analyses by sex and age in our study were not concerned in previous studies [11,12]. We found CC genotype of rs187084 polymorphism increased the risk of OA among old people (age ≥ 55 years), but found no significant association in the subgroup analysis of sex.

Despite the finding about the potential relationship between TLR-9 rs187084 polymorphism and KOA risk, the present study still has some limitations that merit careful consideration. First, confounding factors such as smoking habit and weight may affect the results. Second, the sample size is relatively small, which might underpower our work. Third, selection bias is unavoidable in this hospital-based case–control study. Finally, there is no further subgroup analysis due to limited clinical information.

In conclusion, *TLR*-9 gene rs187084 polymorphism is associated with an increased risk of KOA, especially among old people (age ≥ 55 years). Nevertheless, this finding should be further evaluated by well-designed studies with larger sample sizes and ethnically diverse populations.

## Abbreviations

BMI: body mass index
CI: confidence interval
HWE: Hardy–Weinberg equilibrium
IL-6: interleukin-6
KEGG: Kyoto Encyclopedia of Genes and Genomes
K–L grading: Kellgren–Lawrence grading
KOA: knee osteoarthritis
LD: linkage disequilibrium
NF-κB: nuclear factor-κB
OR: odds ratios
SLE: systemic lupus erythematous
SNP: single nucleotide polymorphism
TLR-9: toll-like receptor 9
TNF-α: tumor necrosis factor-α
